# Creativity and art therapies to promote healthy aging: A scoping review

**DOI:** 10.3389/fpsyg.2022.906191

**Published:** 2022-09-26

**Authors:** Flavia Galassi, Alessandra Merizzi, Barbara D’Amen, Sara Santini

**Affiliations:** Centre for Socio-Economic Research on Aging, IRCCS INRCA-National Institute of Health and Science on Aging, Ancona, Italy

**Keywords:** art therapies, creativity, healthy aging, older adults, prevention, mental health

## Abstract

The purpose of this scoping review is to investigate the value of creative arts therapies in healthy older adults. This article aims to shed light on current knowledge concerning the effectiveness of art therapies (ATs) for the prevention of common age-related conditions using the definition of art therapy provided by the American Art Therapy Association (AATA), as well as Cohen’s conceptual framework for the psychological conceptualization of the relationship between the arts and health in later life. The objective is to carefully capture subthreshold situations of distress, which are often not taken into account and primarily involve psychological aspects that are crucial in the multidimensional perspective of healthy aging. Twelve articles were selected and examined following an initial electronic search on 3 databases. A thematic analysis of the results identified four major themes: improving cognitive performance and proprioception; enhancing self-identity and meaningful life; reducing feelings of loneliness and depressive symptoms; and the importance of socialization. All these aspects constitute the basis for preventing psychological distress and enhancing mental well-being for healthy aging.

## Introduction

The percentage of older adults is projected to nearly double between 2015 and 2050, from about 12 to 22% of the global population (World Health Organization, 2021). Aging of the population causes an increase in multimorbidity (OECD, 2020). Beyond physical ailments, older age is associated with a higher risk of mental diseases (Jokela et al., 2013), the most prevalent of which is depression: a study identified dimensional depression and lifetime major depression as the most prevalent mental health disorders in later life (Volkert et al., 2013).

The onset of mental health problems, such as depressive symptoms and emotional distress, may also coincide with very common existential events, such as the transition from work to retirement (Lucas et al., 2017), or as a reaction to adverse life events, such as the bereavement of a spouse (Fried et al., 2015). Depression is also linked to physical health. For instance, older adults with physical health concerns such as heart disease have higher rates of depression than healthy older adults (Fiske et al., 2009). Untreated depression in an older person suffering from heart disease can have detrimental effects on the individual’s physical health and well-being (World Health Organization, 2017; Hazell et al., 2019). Recent studies have also demonstrated that depression can increase the risk of developing dementia (Hazell et al., 2019; Cantón-Habas et al., 2020). Acting on the early symptoms of depression and mental distress may reduce the risk of developing early cognitive impairment. Although fairly prevalent, depression in older adults is often disregarded by both healthcare professionals and older adults themselves, with the latter receiving psychotherapy far less frequently than younger people (Jokela et al., 2013). In fact, the stigma associated with mental health issues generally discourages the current generation of older adults from seeking assistance. Mental health is a determinant of healthy aging (Jeste et al., 2022). Therefore, from a preventive perspective, its promotion can help older adults lead a meaningful and fulfilling life, particularly through early interventions for initial depressive symptoms (World Health Organization, 2020).

The literature suggests that psychosocial (non-pharmacological) interventions can help improve older adults’ mental health (Chen et al., 2021). In primary care, bibliotherapy, life review, problem-solving therapy, and cognitive behavioral exercise treatments are available for the treatment of late-life depression (Holvast et al., 2017; Chen et al., 2021). Since the late 1930s, art therapy (AT) has been recognized as an intervention for mental health patients in America and the United Kingdom (Malchiodi, 2006; Stuckey and Nobel, 2010; Fancourt and Finn, 2019; American Art Therapy Association, 2021).

Moreover, the potential for creativity and expression was recently incorporated into the gerontology and social science concepts of aging. In fact, older individuals who are unfettered by choices and responsibilities can make room in their lives for self-expression, self-identity, and creativity (Erikson, 1959; Cohen, 2000). This perspective can have a significant impact on research and the conceptualization of the relationship between the arts and health in later life.

### Background

According to the American Art Therapy Association (AATA; American Art Therapy Association, 2021), art therapy, facilitated by a fully trained art therapist, is a treatment option used in ongoing sessions to “improve cognitive and sensorimotor functions, foster self-esteem and self-awareness, cultivate emotional resilience, promote insight, enhance social skills, reduce and resolve conflicts and distress, and advance societal and ecological change.” The AATA adds that, through integrative methods, AT engages the mind, body, and spirit in ways that are distinct from verbal articulation alone. Kinesthetic, sensory, perceptual, and symbolic opportunities open the door to alternative modes of receptive and expressive communication, which can circumvent the limitations of language. Visual and symbolic expressions give voice to experience and empower individual, communal, and societal transformation. According to the AATA, AT is a type of therapy that enhances mental health through “active art-making, creative process, applied psychological theory, and human experience.”

The goal of ATs is to improve or restore the person’s functioning and sense of personal well-being (American Art Therapy Association, 2021). Recent scientific literature has demonstrated that the use of artistic media in healthcare can have lasting benefits on health outcomes. The arts can influence the social determinants of health, encourage health-promoting behaviors, aid in the prevention of health issues, and support caregiving. They can also reduce stress, which helps prevent or slow the progression of a range of conditions, including cardiovascular diseases (Stuckey and Nobel, 2010; Fancourt and Finn, 2019). Creating and experiencing the arts can have profound effects on those afflicted by mental illness. Their ability to provide cognitive stimulation is effective in treating dementia and other age-related conditions (Deshmukh et al., 2018). Art as a means of emotional processing can be effective in the treatment of depression and anxiety (Abbing et al., 2019).

Furthermore, the social interaction associated with the practice of the arts can be an effective way to prevent mental illness risk factors, including loneliness, discrimination, and diminished social capital. Social capital is defined as the networks of relationships among people who live and work in a particular society, enabling that society to function effectively (Fancourt and Finn, 2019).

According to Carr and Hass-Cohen (2008), creative expression and ATs in the field of gerontology can promote healthy aging by fostering a sense of control and the development of positive emotions that can influence physical health, brain plasticity, sense of control mechanisms, and social engagement, as briefly described below.

*Influence of the mind on physical health.* The field of study that helps us understand brain–body relationships is called psychoneuroimmunology (PNI) and refers to the influence of the mind, as mediated through the brain or central nervous system, on the body or immune system (Kiecolt-Glaser et al., 2002a). Based on their studies (Kiecolt-Glaser et al., 2002b) on the effects of positive emotions on the immune system, PNI scientists believe that the positive feelings associated with a sense of control trigger a response in the brain that sends a signal to the immune system to produce more beneficial immune system cells.

*Brain plasticity.* The field of behavioral neuroscience has revolutionized the way we understand the brain’s ability to adapt and remain vital, which is referred to as brain plasticity (Kramer et al., 2004). The use of colors, gestures, and materials stimulate areas of the brain located within the limbic or emotions system, and particularly the hippocampus, which is responsible for the formation of new brain cells (Stern, 2009). With targeted stimulation, the density and mass of the hippocampus may be increased or preserved, thereby continuing neurogenesis well into old age (Stern, 2009). Therefore, art therapists have initiated the development of a neurobiological framework for AT theory and practice.

*Sense of control mechanism.* The arts provide some of the best opportunities for experiencing a new sense of control or mastery. The arts present unlimited opportunities to create something new and beautiful, while simultaneously providing an enormous sense of satisfaction and empowerment.

*Social engagement.* As a mechanism for promoting health, a growing number of studies (Bassuk et al., 1999; Hebblethwaite et al., 2021) have indicated that social engagement in later life has a positive influence on general health and reduces mortality (Avlund et al., 1998). Many forms of art provide significant opportunities for social engagement, including chorales, poetry groups, bands and other instrumental groups, and groups that engage in painting, writing, drama, and dance.

### The purpose of the scoping review

Many studies have proved that the use of AT interventions can improve older adults’ perceptions of health, well-being, and quality of life, consequently reducing the risk of depression and physical and cognitive decline (Im and Lee, 2014; Van Lith, 2016).

However, the majority of the literature focuses on older adults with pre-existing illnesses, and just a few studies have examined the potential of creativity and the arts as a means of preventing mental illness in older adults who live independently in the community. According to the Arksey and O’Malley (2005) framework, the first step in conducting a scoping review is to define the research questions. Therefore, the questions that guided this review are: (1) what are the effects of AT interventions on the independent elderly population? And (2) in what ways do they promote healthy aging? Advancing on previous studies and literature reviews on ATs, this work aims to investigate AT interventions driven by the multi-dimensional healthy aging paradigm (World Health Organization, 2020) to prevent health disorders and improve quality of life for older adults (average age of 60 years or older, as defined by the WHO; Van Lith, 2016; World health Organization, 2022) who have no diagnosed pathologies significantly impacting everyday living and are neither hospitalized nor residing in care facilities.

## Materials and methods

As outlined in Arksey and O’Malley (2005) framework, the methodology of this scoping review is based on the following stages: (1) define the research question; (2) identify the relevant literature; (3) select the studies; (4) map out the data; and (5) summarize, synthesize, and report the results. The findings of each stage are described in this paper’s corresponding section.

### Eligibility criteria and search strategy

Since we make reference to the concept of prevention, we included quantitative and qualitative studies based on AT interventions on community-dwelling older people without conditions that severely impair daily independence, such as Alzheimer’s disease and Parkinson’s disease. Conversely, we included chronic diseases that are not in an acute phase and are controlled, such as diabetes and cardiovascular disease. The first and third authors conducted an electronic database search on February 9, 2021 using PubMed, ProQuest—Psychology Database, CINAHL Complete—EBSCOHost, to find research publications focusing on the application of ATs and their potential to promote the well-being of older adults. After conducting a pilot search in the selected databases, minor adjustments were made to correct search terms. Finally, a combination of Boolean operator and key terms comprising free terms was applied to the literature search, as shown in Table 1.

**Table 1:** Search criteria in different database.

KEYWORDS/ DATABASE	PUBMED	ProQuest – Psychology Database	CINAHL Complete – EBSCOHost
art therap* AND older adults	“title/abstract”	“abstract”	“abstract”
art therap* AND older people	“title/abstract”	“abstract”	“abstract”
art therap* AND healthy ag*	“title/abstract”	“abstract”	“abstract”
art therap* AND ICT solution*	“title/abstract”	“abstract”	“abstract”
art therap* AND virtual coach*	“title/abstract”	“abstract”	“abstract”
art therap* AND digital coach*	“title/abstract”	“abstract”	“abstract”
creativ* AND ICT solution*	“title/abstract”	“abstract”	“abstract”
creativ* AND virtual coach*	“title/abstract”	“abstract”	“abstract”
creativ*AND digital coach*	“title/abstract”	“abstract”	“abstract”
creativ* AND older adults	“title/abstract”	“abstract”	“abstract”
creativ* AND older people	“title/abstract”	“abstract”	“abstract”
creativ* AND healthy ag*	“title/abstract”	“abstract”	“abstract”

The word followed by an asterisk (*) is used for searching for all terms that begin with the related specif word.

Based on the PRISMA extension for scoping reviews (Tricco et al., 2018) and the search strategy, a total of 1,422 articles were identified through database searches, and 537 duplicates were manually identified and removed. Five different eligibility criteria were implemented for the article selection process. First, only research papers were considered; review articles, dissertations, and position papers were excluded. This was related to the objective of this scoping review, which sought to investigate evidence-based experience of AT-driven studies and their effectiveness in reducing the risk of depression and other mental health issues and promoting healthy aging in older adults. Additional selection criteria were centered on the selected methodological approach, which had to be based on ATs and focused on a psychological theoretical framework. Moreover, specific criteria were related to the subjects’ characteristics, that is, an average age of 60 years or older, no chronic or specific pathologies severely affecting everyday living, and not hospitalized or in care or nursing homes. Younger subjects or non-age-defined target groups were excluded. Finally, this scoping review only included articles written in English.

### Data collection and extraction

The first, second, and third authors chose 885 articles by title and abstract, following each author’s individual selection process. The first author’s screening process was checked by the second to verify the accuracy of the selection process described in the PRISMA chart (Moher et al., 2009; see Figure 1). Each author’s results were consistent with those of the other authors once the eligibility criteria were applied.

**Figure 1:** The PRISMA flow chart for reporting the study screening process.

### Review of studies

Article selection based on full-text reading was simultaneously conducted in the three different databases by the first three authors. All full texts were then reviewed by the first author, who also performed a thematic analysis of the included articles and shared them with the co-authors for re-reading and content flow arrangement. They were subsequently shared with the final author, who provided an independent evaluation and oversight. Data analysis led to the identification of central themes through a process of inductive thematic content analysis (Braun and Clarke, 2006). The authors read the articles in order to find specific meanings and common patterns in the use of ATs and intervention outcomes, from which they constructed initial “codes” that were then categorized based on their similarities. The latter were categorized into themes as described in Table 2.

**Table 2:** Selected studies by purpose and method.

Authors, Year	Country	Sample size	Study purpose	Research method	Intervention model
Greaves and Farbus (2006)	UK	172 participants at baseline; 72 at 6 months and 51 at 12 months	Evaluate a complex intervention for addressing social isolation in older people	Quant-qualitative	*Upstream Healthy Living Centre with the use of mentors. A wide range of activities are provided: painting, print making, creative writing, tai chi, reminiscence, music*
				Qualitative tools	
				– Semi-structured individual interview with 26 participants, 5 careers and 4 health professionals	
				– Focus groups	
				Quantitative measures used: Geriatric Depression Scale; SF12 Health Quality of Life; Medical Outcomes Social Support Scale	
Marmeleira et al. (2009)	Portugal	37 older people (divided in experimental and a control group)	Investigate the effects of a creative dance program on proprioception of older adults	Quantitative, pre-post studio: (inter-group and intra-group analysis)	12-week *creative dance program* (3 sessions of 90 min per week)
				– knee proprioception assessed through JPS	
				– kinesthesia assessed through Biodex System 2 12 weeks follow-up	
Pitkala et al. (2011)	Finland	235 older people	Determine the effects of socially stimulating group intervention on cognition among older individuals suffering from loneliness	Quantitative/longitudinal (baseline-at three months-after one year)	(1) *Art, inspiring activities and discussion,* (2) *Exercise and nature and discussion,* (3) *Therapeutic writing and discussion*
				– Charlson comorbidity index	
				– MMSE	
				– CDR	
				– ADAS-Cog and HRQoL	
Alders Pike (2013)	Miami-Florida	91 older adults	Examine the effect of 10-week AT intervention on the cognitive performance among a moderate size, ethnically diverse sample of older adults	Quantitative/pre-post test	*Ad hoc* designed *AT protocol*: 10-week intervention
				– Clock Drawing Test (CDT)	
				– Cognitive Failures Questionnaire (CFQ)	
Stephenson (2013)	USA	70 older people (Divided in groups of 10 to 15 participants)	Longitudinal evaluation of the CATS program over 6 years, in:	Qualitative assessment: shared discussion about the artwork created	*Open, non-directive, AT studio* (groups that met weekly for 2 h)
			(1) foster artistic identity		
			(2) activate a sense of purpose and motivation		
			(3) use art as a bridge to connect with others		
			(4) support movement toward the attainment of gerotranscendence		
Engelbrecht and Shoemark (2015)	Australia	5 community-dwelling older women	Investigate the acceptability and efficacy of using iPads in music therapy intervention compared to traditional music instruments	Pre-post intervention	*Music therapy mediated by technology*: 5 60-min sessions of music therapy
				Qualitative: – Journal entry (after each session)	
				Quantitative: – Friendship scale − Rosenberg self-esteem scale	
Ilali et al. (2018)	USA	54 older people	Evaluate the impact of a drawing-based life review program on reducing depression symptoms	Quantitative/longitudinal: experimental art group and control group demographic questionnaire, AMT screening tool and GDS questionnaire and 2 follow up (1 week later and 1 month later)	Six weekly sessions of the *life review* that is a *specific AT intervention*
Diaz Abrahan et al. (2019)	Argentina	30 older people (divided in experimental group and control group)	Evaluate the effectiveness of music therapy in improving the quality of life of older adults	Quantitative:	Weekly 2-h *music therapy* meetings for a period of 8 months
				– Questionnaire for socio-demographic data	
				– IQoL (inventory of quality of life)	
				– Extra-individual assessments by inventory	
McCarthy et al. (2019)	USA	20 older women (with a normal score at Mini-Cog Dementia Test) divided by 2 groups of 10	Evaluate participants’ experiences of PATH program and the meaning ascribed to those experiences	Qualitative:	Self-transcendence *PATH program* (8-week theory-based intervention) *combining mindfulness exercises, group processes and creative projects reinforced by home practice*
				– Audiovisual recordings	
				– Weekly group discussions and focus groups The data were coded using an inductive approach	
Poulos et al. (2019)	UK-Australia	127 older people	Promote health and well-being. Evaluate the AOP model	Quant-qualitative/pre-posttest	*AOP: participatory art program* (weekly classes for 8–10 weeks) in which are involved healthcare practitioners and professional artists (visual arts, photography, drama, dance and movement, singing and music).
				Quantitative measures: – WEMWBS – CAT: questionnaire for measure the perception of creativity (level and frequency) And measures of frailty with the criteria: unintentional weight loss, exhaustion, low physical activity level, slow walking speed, weakness	
				Qualitative tools (over the program period): – 8 focus groups involving 19 males and 29 female participants – 4 interviews with a predetermined list of questions (recorded and transcribed)	
Malyn et al. (2020)	UK	20 older people	Develop a deeper understanding of the therapeutic mechanism occurring within creative writing groups	Qualitative: thematic analysis of semi-structured individual interviews lasting 40 min and audio-recorded	*Creative writing and bibliotherapy*
Schoales et al. (2020)	Canada	10 older people	Examine wellbeing among older adults while exploring the effects of engaging in a creative digital storytelling workshop	Qualitative: one-on-one semi-structured interviews that last from 30 to 90 min, interpretive phenomenological inquiry	*Creative digital 3-day storytelling workshop*

## Results

### Description of selected studies

The search returned 885 results. Following the elimination of 760 articles based on the analysis of titles and abstracts, the remaining 125 full articles were assessed for eligibility. This selection process culminated in the final inclusion of 12 eligible articles (see Figure 1).

In accordance with the framework proposed by Arksey and O’Malley (2005); Table 2 provides an overview of the selected studies, which are discussed in more detail below. The earliest study was conducted in the United Kingdom in 2006, while the most recent article, which was also conducted in the United Kingdom, was published in 2020. More than half of the selected studies are from the Americas, including four from the United States, one from Argentina, and one from Canada. Two studies are Australian. Finally, there are five European studies, including three from the United Kingdom, one from Finland, and one from Portugal. The selected articles have different sample sizes, ranging from 5 to 235 individuals, based on the adopted research methodology. Only McCarthy et al. (2019) focused on one-gender participants, with 20 women in their study, while all the other studies included both women and men. The selected articles were based on studies that evaluated the impact of different types of ATs on general life domains such as health and well-being (Poulos et al., 2019), quality of life (Diaz Abrahan et al., 2019; Malyn et al., 2020), and the general arts experiences (McCarthy et al., 2019), or specific sub-domains such as social isolation (Greaves and Farbus, 2006) and proprioception (Marmeleira et al., 2009). Other sub-domains are cognition (Pitkala et al., 2011; Alders Pike, 2013), motivation (Stephenson, 2013), and depression (Ilali et al., 2018).

In terms of the research method, four studies adopted a qualitative method (Engelbrecht and Shoemark, 2015; Ilali et al., 2018; McCarthy et al., 2019; Malyn et al., 2020), five a quantitative approach (Marmeleira et al., 2009; Alders Pike, 2013; Stephenson, 2013; Ilali et al., 2018; Diaz Abrahan et al., 2019), and three a quant-qual methodology (Greaves and Farbus, 2006; Engelbrecht and Shoemark, 2015; Poulos et al., 2019). Seven studies included a pre-post assessment or one or two follow-ups (Greaves and Farbus, 2006; Marmeleira et al., 2009; Pitkala et al., 2011; Alders Pike, 2013; Stephenson, 2013; Engelbrecht and Shoemark, 2015; Ilali et al., 2018; Poulos et al., 2019; Schoales et al., 2020). The studies involved different interventions.

Four of the studies included multiple types of ATs (Greaves and Farbus, 2006; Pitkala et al., 2011; McCarthy et al., 2019; Poulos et al., 2019). The other studies are more specific in terms of the type of AT used: one study discusses creative writing (Malyn et al., 2020), two studies focus on AT and its therapeutic models (detailed below; Stephenson, 2013; Ilali et al., 2018), two studies discuss music therapy (Engelbrecht and Shoemark, 2015; Diaz Abrahan et al., 2019), one study discusses creative dance (Marmeleira et al., 2009), and one study focuses on digital storytelling (Schoales et al., 2020). The AT interventions described in the selected studies last between a minimum of 2 months to a year or more, except for the digital storytelling intervention (a three-day workshop; Schoales et al., 2020) and the five one-hour sessions of technology-mediated music therapy (Engelbrecht and Shoemark, 2015). The studies are listed in Table 2 in chronological order; however, for the sake of logic and clarity of presentation, we will discuss them on the basis of the intervention methodology employed.

### Multimethod studies

McCarthy and colleagues (McCarthy et al., 2019) applied and examined the Psychoeducational Approach to Transcendence and Health (PATH) program by engaging 20 older women in an 8-week theory-based intervention combining mindfulness exercises, group processes, and creative projects reinforced by home practice. The program is based on Reed’s self-transcendence theory (Reed, 2018). Self-transcendence is a developmental process inherent in later life that shapes one’s perspective on self, others, the material world, and the spiritual or existential dimension. In the older adult population, self-transcendence has been associated with well-being, meaning in life, hope and transcending loss, decreased depression, resilience, sense of coherence and purpose in life, inner strength, flexibility and creativity, more satisfying social relationships, improved physical and mental health, and improved self-care.

The Art on Prescription (AOP) Model evaluated by Poulos et al. (2019) reflects the international shift from the biomedical model of health to a more holistic approach, which sees health as “complete physical, mental, and social well-being” (Rigby, 2004). In this study, conducted in Sydney, Australia, 127 older adults were referred to the program by their healthcare practitioners. Professional artists led courses in visual art, photography, dance and movement, drama, singing, or music with the aim of aiding recovery and promoting healthy aging. A pre-post quantitative and qualitative evaluation was carried out. Quantitative assessments included the Warwick-Edinburgh Mental Well Being Scale (WEMWBS; Tennant et al., 2007) and a common assessment tool (CAT) developed *ad hoc* for the study, which incorporated measures of frailty.

Focus groups and individual interview topic guides were used as qualitative tools.

The Upstream model adopted by Greaves and Farbus (2006) is a complex intervention for preventing social isolation and depression in older people. The model promotes active social contact (McAuley et al., 2000), encourages creativity (Smith and Andersson, 1989), and uses mentoring (Bennetts, 2000). A wide range of activities were provided: painting, printmaking, creative writing, Tai Chi, reminiscence, music, and others, in a vast study that involved 172 participants at baseline, 72 at 6 months, and 51 at 12 months. The model was evaluated by using both quantitative [e.g., Geriatric Depression Scale (Sheikh and Yesavage, 1986); SF12 Health Quality of Life (Huo et al., 2018); Medical Outcomes Study Social Support Scale (Sherbourne and Stewart, 1991)] and qualitative measures (semi-structured individual interviews with 26 participants, 5 careers, and 4 health professionals and focus groups).

Pitkala et al. (2011) selected a very large sample of 235 lonely older adults for a psychosocial group intervention that included art and stimulating activities, exercise and nature, therapeutic writing, and a verbal discussion at the conclusion of each meeting. The group leaders were nurses, occupational therapists, or physiotherapists who had received detailed training (Pitkala et al., 2004). To investigate the cognitive effects of socially stimulating group therapies, this study used the following tools at baseline, 3 months, and after 1 year: the Charlson comorbidity index (Charlson et al., 1987), which takes into account the number and severity of comorbid conditions; the Mini Mental State (MMSE; Folstein et al., 1975); CDR (Hughes et al., 1982), which is a clinical scale for identifying the stage of cognitive impairment or dementia; the ADAS-Cog (Rosen et al., 1984), which consists of a set of brief neuropsychological evaluation tools used to assess the severity of dementia cognitive symptoms; and the 15D measure (Sintonen, 2001) that is a generic, comprehensive, 15-dimensional, standardized, self-administered measure of health-related quality of life (HRQoL).

### Art therapy studies

The Alders Pike (2013) study examined the effects of 10 weeks of AT on cognitive performance in a moderate-sized, ethnically diverse sample of 91 older adults. In this experience, cognitive training strategies served as a framework, and a specific protocol was used and implemented by all the art therapists involved, employing a pre and post-test design and utilizing the Clock Drawing Test (CDT; Nishiwaki et al., 2004) and the Cognitive Failures Questionnaire (CFQ; Wagle et al., 1999).

The Stephenson (2013) study reported the results of a program based on the Creative Aging Therapeutic Services (CATS), which forms part of a longitudinal community program founded on the belief that art-making can be a meaningful and important component of aging well, as framed by Tornstam’s theory of gerotranscendence (Tornstam, 2005). Seventy older adults participated in an open, non-directive AT art studio for 6 years (Finkel and Bat Or, 2020). Participants shared their thoughts, ideas, and feelings regarding their own artwork and the artwork of other participants at weekly group meetings.

There was no mention of whether the group discussions were guided by a topic, of who moderated the sessions, or how the content was analyzed. Ilali et al. (2018) investigated the impact of an AT-based life review process on depressive symptoms in a sample of 54 older adults. This technique can be employed as a primary, evidence-based treatment for depression in later life (Korte et al., 2012). The life review’s therapeutic aspect appears to be the revival of memories of past experiences and conflicts, which can lead to reassessment, identification of solutions, and the possibility of the individual’s improved coherence and sense of integrity. A life review is typically structured around one or more family-centered life themes, ranging from a person’s childhood to their experience as a parent or grandparent (Haber, 2006).

### Music therapy studies

The study by Diaz Abrahan et al. (2019) assessed the impact of weekly music therapy meetings on a group of 30 older adults as a non-pharmacological strategy to improve older people’s quality of life in order to promote healthy aging or prevent pathological aging.

The pre-post intervention study conducted by Engelbrecht and Shoemark (2015) on five community-dwelling older women explored the acceptability and efficacy of using iPads as opposed to traditional music instruments to administer music therapy. They used both qualitative and quantitative tools, such as diary writing (Jacelon and Imperio, 2005), the Friendship Scale to quantify older people’s social isolation (Hawthorne, 2006), and the Rosenberg Self-Esteem Scale (Rosenberg, 1965).

### Creative dance study

Marmeleira et al. (2009) measured knee proprioception and kinesthesia with the Joint Position Sense (JPS; Riemann et al., 2002) and Biodex System 2 (Biodex Medical Systems, Shirley, New York) to assess the impact of a 12-month creative dance program on proprioception in a group of 37 older adults. In this study, creative dance is defined as a particular form of dance that does not require years of training and lacks predetermined performance standards (Lewis and Scannell, 1995).

### Creative writing and digital storytelling studies

Malyn et al. (2020) implemented a program that focused on community-based bibliotherapy and therapeutic creative writing groups. Four overarching themes concerning the relationship with the self, with others, with facilitators, and with an intermediary object emerged from the qualitative analysis of the interviews with the 20 participants. The study by Schoales et al. (2020) relied on the technique of creative digital storytelling with the use of technology, and involved 10 individuals who had participated in a three-day digital storytelling workshop. Van Manen (2014) conducted qualitative interviews using interpretative phenomenological inquiry to assess the well-being of 10 participants.

### Thematic analysis of the studies

In addition to the common and overarching goal of improving the well-being and quality of life of older adults, four main themes emerged from the analysis of the results obtained from the various AT-mediated interventions: improving cognitive function and proprioception; enhancing self-identity and a meaningful existence; reducing depression and a sense of loneliness; and the importance of socialization. Tabulated in Table 3 are the studies grouped by their findings’ main themes and sub-themes.

**Table 3:** Theme and sub-themes (when applicable) within selected articles.

Main themes	Sub-themes	Studies reference
1. Cognitive performance and proprioception	Cognitive performance improvement Therapeutic approach employed by therapist, along with the duration of treatment, positively affected cognitive performance; Longer sessions and a combined approach of “art as therapy” and art psychotherapy correlate with better performance	Alders Pike, 2013
	Proprioception improvement Creative dance program emphasizing body awareness	Marmeleira et al., 2009
	Improved mental function Decreased lonely	Pitkala et al., 2011
2. Self-identity and meaningful life	Self-image improvement A new perspective of life and death Personal meaning in past experiences Positive self-identities	McCarthy et al., 2019
	Improved well-being	Malyn et al., 2020
	Quality of life improvement Music therapy	Diaz Abrahan et al., 2019
	Improved sense of purpose and motivation Improved socialisation use art as a bridge to connect with others Gerotranscendence	Stephenson, 2013
	Improved mental well-being Improved sense of purpose Personal growth and achievement Empowering Enhanced interpersonal relationships	Schoales et al., 2020
3. Reducing loneliness and symptoms of depression	Depression decrease Ego-integrity improvement Depression prevention	Ilali et al., 2018
	Effectiveness of digital technology to use in music therapy with older people	Engelbrecht and Shoemark, 2015
4. The importance of socialization	Upstream model Social networks Psychosocial and health benefits A reversal of the expected downward trends in some aspects of participants’ health	Greaves and Farbus, 2006
	Improved individual well-being Enjoyment Efficacy Relationships	Poulos et al., 2019

#### Cognitive performance and proprioception

The Alders Pike (2013) study is the first to examine this topic; it demonstrates that cognitive performance can improve after a 10-week program of AT sessions. The findings indicate that the AT approach and the length of treatment positively impacted cognitive performance; and finally, longer sessions and a combined approach of “art as therapy” and art psychotherapy are associated with improved performance. The creative dance program evaluated by Marmeleira et al. (2009) is in the same thematic group. This study demonstrated that body awareness can improve proprioception, which can provide a unique sensory component to optimize motor control. Its importance in older adults has been consistently reported in terms of balance, walking stability and trajectory, sit-to-stand performance, and stair-climbing ability (Lord et al., 2002). Creative dance further amplifies these effects by stimulating creativity through a positive learning environment and adding extra dimensions, such as an individual’s self-mastery, by allowing the subjects to be consciously aware of their bodies. The study by Pitkala et al. (2011) is the first randomized controlled trial to demonstrate that art and inspirational activities, such as therapeutic writing, significantly improved the cognition of lonely older adults in the intervention group in comparison to the control group, which received conventional cognitive training.

#### Self-identity and a meaningful life

Five studies observed the influence of ATs on the self-identity and meaningfulness of individuals’ lives (Stephenson, 2013; Diaz Abrahan et al., 2019; McCarthy et al., 2019; Poulos et al., 2019; Malyn et al., 2020). The 20 women who participated in the PATH program assessed by McCarthy et al. (2019) gained a new perspective on life and death; they identified personal meaning in past experiences and were supported in developing a positive sense of self. Participants in the AOP intervention delivered by Poulos et al. (2019) reported a statistically significant improvement in the results of mental well-being, as measured by the WEMWBS (Warwick-Edinburgh Mental Well Being Scale) and self-reported creativity. Moreover, the AOP provided participants with a sense of purpose and direction, facilitated personal growth and achievement, and empowered them to form meaningful relationships with others. Malyn et al. (2020) concluded that the therapy promotes the well-being of older adults by creating a unique environment in which participants feel acknowledged, accepted, challenged, and inspired. The study by Diaz Abrahan et al. (2019) also demonstrates AT’s positive effects on the meaning of life. In fact, older adults who attended weekly music therapy meetings scored higher on the inventory of quality of life (IQoL) and its subcomponents (religion, creativity, recreation, and love) in terms of total quality of life. The research conducted by Stephenson (2013) demonstrated that the AT program can stimulate artistic identity and activate a sense of purpose and motivation in participants through creative work. Furthermore, this study proved that the use of art can facilitate human connection and promote gerotransendence.

#### Reducing feelings of loneliness and symptoms of depression

The study by Ilali et al. (2018), conducted in the United States, analyzes the impact of a drawing-based life review program on depressive symptoms in a sample of 54 older adults. This technique can be employed as a primary, evidence-based treatment for depression in later life (Erikson, 1959). This study demonstrates that after a six-week drawing-based life review intervention, the experimental group’s depressive symptoms decreased and the older adults’ ego integrity improved, thus preventing depression and despair, and the structure of group sessions appeared effective at reducing depressive symptoms. Finally, the study by Engelbrecht and Shoemark (2015), which targeted the health risk factors of social isolation and low self-esteem in a group of five community-dwelling women, demonstrates that technology can be an acceptable and potentially successful tool for use in music therapy with older adults.

#### The importance of socialization

The research conducted by Greaves and Farbus (2006) reveals that the Upstream Model generates social networks, a range of psychosocial and health benefits, and a reversal of expected downward trends in certain aspects of participants’ health. The key outcomes were the formation of a positive group identity and the enhancement of participants’ self-confidence and self-efficacy. Similarly, Schoales et al. (2020) found that group AT programs can generate enjoyment and social ties, which can amplify the effects of ATs on individuals’ well-being.

The themes that emerged from the analysis are similar to the Positive Emotion, Engagement, Relationships, Meaning, and Accomplishment (PERMA) model (Seligman, 2011), which draws on both pleasure-focused hedonic factors and eudemonic elements that emphasize moral development and self-growth. The findings of these two studies demonstrate that the development of a positive group identity and socialization within AT workshops and activities can boost confidence and self-efficacy.

## Discussion

### Advances in the knowledge of art therapies as a means of promoting healthy aging

This review’s main novelty is its focus on studies reporting the outcomes of AT interventions targeting independent community-dwelling older adults from a preventive standpoint. This study’s thematic analysis provided evidence of the efficacy of ATs in promoting cognitive functions (Marmeleira et al., 2009; Pitkala et al., 2011; Alders Pike, 2013), mental well-being (by fostering self-identity, self-efficacy, and by reducing depressive symptoms; Stephenson, 2013; Engelbrecht and Shoemark, 2015; Ilali et al., 2018; Diaz Abrahan et al., 2019; McCarthy et al., 2019; Malyn et al., 2020; Schoales et al., 2020), and socialization (Greaves and Farbus, 2006; Poulos et al., 2019), all of which can be considered psychological dimensions of healthy aging and preventive aspects of depression (World Health Organization, 2017, 2020).

Thus, the analysis supports and corroborates current knowledge on creativity and ATs as tools to enhance personal feelings of well-being and key physiological and psychological functions such as cognition, emotions, and proprioception (Carr and Hass-Cohen, 2008). More specifically, ATs can play a pivotal role in the delivery of health and social care interventions to promote healthy aging among older adults (World Health Organization, 2017).

Even though the reviewed studies investigated the efficacy of ATs on specific well-being domains, Carr and Hass-Cohen (2008) framework states that all these aspects should be considered interconnected because they all contribute to psychological well-being and can help prevent the most common age-related pathologies, such as Alzheimer’s disease and other dementias (Deshmukh et al., 2018; Fancourt and Finn, 2019). Our findings are comparable with those of several other studies indicating that engagement in an environment enriched with creative materials and stimulation from ATs may foster neurogenesis (increased production of new neurons). Indeed, this type of environment encourages physical activity (e.g., by manually creating a drawing or a sculpture), problem solving (e.g., by choosing colors or compositional elements), and socialization (e.g., by creating, sharing, and describing one’s artwork in a group; Bassuk et al., 1999).

The results also highlight the importance of the group dimension in the execution of AT programs. Artistic and expressive group activities appear to stimulate socialization, which, in turn, mitigates the perception of loneliness and depressive symptoms, when present (Hocoy, 2002). This review validated current knowledge regarding the effectiveness of ATs in enhancing healthy aging, particularly mental well-being and socialization, among older adults living independently, and shed light on the potential of ATs to prevent age-related diseases (Fiske et al., 2009; Jokela et al., 2013; World Health Organization, 2017; Barnes et al., 2021).

### Critical aspects and insights related to the topic

This scoping review also uncovered certain critical aspects. One such aspect lies in the very definition of AT, which is not unique and multifaceted. In fact, as defined by the British Association of Art Therapist (BAAT), AT is a form of psychotherapy that uses art media as its primary mode of communication. Clients who are referred to an art therapist need not have experience or skill in art. The art therapist is not primarily concerned with making an aesthetic or diagnostic assessment of the client’s image. The overall aim of its practitioners is to enable a client to change and grow on a personal level through the use of art materials in a safe and facilitating environment. AT is not a recreational activity or an art lesson, although the sessions can be enjoyable. Clients do not need to have any previous experience or expertise in art.

Moreover, from a literature review commissioned by the Psychotherapy and Counselling Federation of Australia (PACFA; Dunphy et al., 2013) the terms “expressive arts therapy” and “creative arts therapy” were found to be used interchangeably, referring to the overall practice of the arts applied as therapy. “Expressive arts therapy” is more common in European practice, while “creative arts therapy” is more frequently used in Australia. Both terms can also refer to a multi-modal approach wherein a therapist employs a range of art forms as an integral aspect of their practice. One of the most accurate definitions might be that given by the Australian and New Zealand Arts Therapy Association (ANZACATA, 2012), according to which Arts therapy or arts psychotherapy is a form of psychotherapy that uses creative modalities, including visual art-making, drama, and dance/movement to improve and inform physical, mental and emotional well-being. Arts therapy works by accessing imagination and creativity, which can generate new models of living, and contribute towards the development of a more integrated sense of self, with increased self- awareness and acceptance.

In reality, there are numerous approaches that we have attempted to include in a single theoretical framework by primarily referring to the AATA definition (American Art Therapy Association, 2021), that we felt was most suitable and inclusive, and by making certain choices: we excluded all activities considered to be merely recreational and, in the AT container, we included all forms of creative expression treated from a therapeutic perspective, such as painting, sculpture, drawing, dance, creative writing, and music. Another point of reflection concerns who conducts AT experiences and how they do so. If we take the AATA website as a reference, art therapists are described as “master-level clinicians who work with people of all ages across a broad spectrum of practices.” Guided by ethical standards and scope of practice, their supervised education and training prepares them for culturally competent work with diverse populations in a variety of settings.

Art therapists work with people facing medical and mental health issues, as well as individuals seeking emotional, creative, and spiritual growth (American Art Therapy Association, 2021). Following the BAAT definition we go on to say that Art therapists have a good understanding of art processes, underpinned by a sound knowledge of therapeutic practice, and work with individuals and groups in a variety of residential and community based settings. Although influenced by psychoanalysis, art therapists have been inspired by theories such as attachment-based psychotherapy and have developed a broad range of client-centred approaches such as psycho-educational, mindfulness and mentalization-based treatments, compassion-focused and cognitive analytic therapies, and socially engaged practice. Exploring the links between neuro-science and art therapy has also been at the forefront of some of the BAAT’s conferences. Importantly, art therapy practice has evolved to reflect the cultural and social diversity of the people who engage in it.

However, the selected articles contain different approaches. With the exception of one study, which focuses on the role of the therapist and the importance of sufficient training for effective therapeutic interventions (Pitkala et al., 2011), the level or type of therapist training is frequently not well-defined (Marmeleira et al., 2009; Diaz Abrahan et al., 2019; Schoales et al., 2020). Sometimes, the therapist is a mentor or facilitator who is given specific instructions (Greaves and Farbus, 2006; Malyn et al., 2020); or a nurse, psychologist, or occupational therapist who has received specific training in AT (Pitkala et al., 2011; Ilali et al., 2018; McCarthy et al., 2019); or a professional artist (Schoales et al., 2020); or even art therapists who are university graduates (Alders Pike, 2013; Stephenson, 2013). In reality, AT training is open to many different professionals in different countries, so it is possible to find art therapists with different backgrounds and training of different durations and with different curricula. AT programs developing around the world need an educational framework to ensure that graduates have a knowledge base and set of skills consistent with peers in other countries. There are currently many independent training standards offered by art therapy associations in the United Kingdom, the United States, Canada, Australia, and New Zealand, United States, Canada, Australia, and New Zealand, as well as two international associations. Research still in press, attempted to synthesize these requirements, revealing 12 content areas that can form the core of art therapy training. Even within these standards, programs developing around the world must consider local values related to health, art, therapy, and education to create globally relevant and locally meaningful art therapy training programs (Potash et al., 2012).

Therefore, it should be emphasized that AT therapists who seek to improve the physical, mental health, and social functioning of older adults must be professionally trained and have the necessary educational background (Dunphy et al., 2019). From this point of view, it would be interesting to devote extra effort to cross-research the educational curricula offered by various professional art therapy associations.

In the context of the healthy aging paradigm (Jeste et al., 2022), the purpose of this review was to identify and highlight the beneficial effects of ATs for the prevention of mental distress, while considering those aspects of mental health that are closely related to physical health and social well-being. We did not, however, delve into the processes (the why) by which ATs accomplish these objectives. Rather, we used the AATA definition, identified the topic areas where the interventions were effective, and presented a discussion that included the quality of the art therapist’s training, the duration, and the grouping of the interventions as critical factors for their success. This and other recent research in the field of ATs (Cohen et al., 2006; Regev and Cohen-Yatziv, 2018; De Witte et al., 2021) have left certain questions unanswered, for instance, why various types of AT interventions are effective and what their neurobiological bases are.

Finally, we found only two articles that implemented hi-tech solutions in ATs for older adults. Given the growing interest in practice and research in this field, it is important to investigate how art therapists engage with digital technology and how (and if) this approach can be safely adapted to encompass new potential ways of delivery and new artistic media (Zubala et al., 2021). This could be especially intriguing in light of the global spread of the SARS-CoV-2 virus, which has opened the doors to the virtual world in the AT field. However, the pros and cons are still unclear, and further research is necessary to determine how to advance the use of ATs to improve older adults’ attitudes toward healthy aging.

### Limitations and suggestions for future research studies

This review is not without its limitations. Several studies may have been overlooked because they were available in languages other than English on search engines that were not accessed during this review, and others may have been published after the search was completed. Another limitation is the stringent study selection criteria. In fact, the goal of identifying only those studies based on AT interventions targeting independent community-dwelling older adults resulted in the inclusion of a small number of articles because the majority of studies on ATs target (older) people with disabilities and/or those attending elderly care facilities.

Moreover, despite the availability of a substantial corpus of “grey literature” on ATs, this review focused exclusively on scientific studies providing evidence-based outcomes. Another limitation is the absence of a consultation exercise which, according to Arksey and O'Malley (2005), is optional but may have made the results more relevant to policymakers, practitioners, and service users. Since the purpose of this review is to map research activities in the AT field, evidence sources were not critically appraised.

It is recommended that future research and reviews specifically focus on one type of intervention, for instance, to learn more about the success factors of music therapy versus dance movement therapy or art therapy. In order to acknowledge that expressive and creative modalities are not limited to drawing alone, but include a variety of non-verbal languages as defined by the AATA (American Art Therapy Association, 2021), we accepted studies employing a wide range of outcome assessment methodologies and included several types of ATs. The gender, educational level, and multiculturalism of participants are other aspects that may be interesting to explore but were not the subject of this review. Only one of the selected studies considered the influence of ethnicity on the effectiveness of the ATs program by including individuals from diverse ethnic and cultural backgrounds (Stephenson, 2013), and none of the studies considered the educational level of participants as a possible factor influencing the effectiveness of ATs.

Given that the studies under consideration were conducted in the United States and Europe, it is reasonable to assume that the positive outcomes of creative activities and art therapies are transcultural and inclusive, permitting both verbal and non-verbal expression through gestures, sounds, graphics, and plastic signs; thus, they can be considered a universal language (Hocoy, 2002). All but two of the samples included male and female participants (Engelbrecht and Shoemark, 2015; McCarthy et al., 2019), revealing that the majority of the selected studies also lacked a gender viewpoint. Given that AT enables the client and therapist to explore issues that are often difficult to articulate in words, and that one such issue is the complexity of gender, it is recommended that future research investigates how cultural and ethnic aspects and gender influence participants’ responses to AT-based interventions, particularly in the aging phase and from the perspective of healthy aging (Hogan, 2002). Therefore, we do not claim to be exhaustive, but we believe that our focus on interventions targeting independent, community-dwelling older adults is the key aspect, necessitating the exclusion of certain elements and facets of the topic’s complexity.

## Conclusion

Art therapists in gerontology have traditionally focused on treating patients with established conditions, such as dementia in general and Alzheimer’s disease in particular (Ozdemir and Akdemir, 2009; Deshmukh et al., 2018). However, it is not inconceivable that they could also play a significant role in promoting healthy aging and preventing or delaying the need for medical intervention. Numerous older adults are at risk of becoming isolated, depressed, or incapable of taking care of their daily needs. Through participation in AT programs, older adults may continue to interact with their peers and communities, and become motivated to lead active lives. AT can boost their self-esteem and provide them with opportunities to develop previously unexplored aspects of their identities. Policymakers, commissioners, and care providers in health and social care must acknowledge that the arts and ATs are not a marginal and elitist avenue, but rather a mainstream tool that helps older people remain active, healthy, and independent. In fact, ATs constitute a powerful source of motivation, agency, and confidence that, when coupled with rigorous methodology for the assessment of outcomes, can provide new advancements for the delivery of measures to delay early cognitive deterioration, depression, and social isolation in older adults.

## Author contributions

FG and SS: conceptualization. FG, BD’A, and SS: methodology. AM, FG, and BD’A: formal analysis. FG and BD: writing—original draft preparation. AM and SS: writing—review and editing. All authors contributed to the article and approved the published version.

## Funding

This study was supported by Ricerca Corrente funding from the Italian Ministry of Health to IRCCS INRCA.

## Conflict of interest

The authors declare that the research was conducted in the absence of any commercial or financial relationships that could be construed as a potential conflict of interest.

## Publisher’s note

All claims expressed in this article are solely those of the authors and do not necessarily represent those of their affiliated organizations, or those of the publisher, the editors and the reviewers. Any product that may be evaluated in this article, or claim that may be made by its manufacturer, is not guaranteed or endorsed by the publisher.
